The article "The Application Effect of Evidence-Based Care in Gastrointestinal Surgical Pipeline Nursing" was retracted in 2023. Reasons: unreliable results or conclusions; lack of ethics approval or compliance; concerns about the data; concerns about the peer review.

# The Application Effect of Evidence-Based Care in Gastrointestinal Surgical Pipeline Nursing

**DOI:** 10.1155/2022/5027024

**Published:** 2022-07-28

**Authors:** Xiaoyan Chen, Qianqian Song, Junhong Wu, Zonglan Fang, Guiyuan Sui

**Affiliations:** ^1^Infection Management Office, Affiliated Hospital of Shandong University of Traditional Chinese Medicine, Jinan, 250014 Shandong, China; ^2^Department of Digestive Endoscopic Diagnosis and Treatment, Affiliated Hospital of Shandong University of Traditional Chinese Medicine, Jinan, 250014 Shandong, China; ^3^Health Care West Ward 15, Affiliated Hospital of Shandong University of Traditional Chinese Medicine, Jinan, 250014 Shandong, China; ^4^Department of Infectious Diseases, Yantai Penglai Hospital of Traditional Chinese Medicine, Penglai, 265600 Shandong, China; ^5^Haemodialysis Room, Affiliated Hospital of Shandong University of Traditional Chinese Medicine, Jinan, 250014 Shandong, China

## Abstract

With the improvement of the higher nursing education system, the overall quality and work ability of clinical nurses have also been significantly improved. Most nursing staff have a positive attitude towards evidence-based nursing medicine but lacking of the knowledge and skills about evidence-based nursing. Clinical nurses are still short of the ability to evaluate relevant research data, which is one of the cause of interference for the clinical nurses to use the latest research results reasonably and effectively at present. The purpose of this paper is to explore the application effect of evidence-based nursing in gastrointestinal surgical pipeline nursing and to clarify the impact of evaluation ability on nurses in clinical practice, investigate, and discuss the application effect of evidence-based nursing in gastrointestinal surgical pipeline nursing. This paper selects the clinical nurses of the three top three hospitals in a province as the research object, using the ways of general data questionnaire, the general individual performance sensitivity scale, the evidence-based nursing application behavior questionnaire, the evidence-based nursing application behavior willingness questionnaire, and the evaluation ability training needs questionnaire to collect data for 100 cases of gastrointestinal surgery clinical nurses. Analyze nurses' awareness level of evidence-based nursing, the willingness of evidence-based nursing behavior, and the relevance of evidence-based nursing behaviors. Use multiple regression analysis methods to explore its influencing factors, and use data statistics to analyze the role and effect of evidence-based nursing in the gastrointestinal surgery pipeline. The research results show that the evaluation ability has a significant promotion effect on clinical nursing application, and it is one of the important factors for clinical nurses to use evidence-based nursing. Clinical nurses have a higher demand for evaluation ability training, and basically here, the application effect of evidence-based nursing in the gastrointestinal surgical pipeline nursing is relatively good.

## 1. Introduction

Personal expression is the confidence of a person's ability to achieve a given ultimate goal. Personal performance perception can be divided into general individual performance perception and special performance perception, and its goal is specific and final [1]. In general, individual performance refers to their overall confidence in facing different end goals. What they express is their self-confidence, whether they can adopt adaptive behavior when facing new things or new challenges. Most of the current research on the clinical performance of clinical nurses is based on general individual performance. As an effective working method and procedure, evidence-based nursing medicine has been highly valued and appreciated by people since its introduction into China [2]. Evidence-based nursing medicine has gradually gained more and more applications in the country. However, the current application of evidence-based nursing in clinical nurses is not satisfactory and is affected by various interference factors [3]. These data can be divided into two categories: the external objective reasons and internal causes of the clinical nurses themselves. In traditional abdominal surgery, nasogastric tube decompression is a normal thing and a recognized rule. In fact, placement of the nasal and gastric tubes can cause very uncomfortable patients, including nausea, vomiting, and mucosal discomfort, and affect early postoperative activities. The placement of the nasal and gastric tubes increases the likelihood of inflammation of the lungs. No nasal and gastric tubes were seen before surgery. Although postoperative abdominal distension and nausea and vomiting were aggravated, the incidence of postoperative throat inflammation, pharyngeal discomfort, and pulmonary inflammation decreased [4]. For example, sometimes, the nasal tube and the stomach tube are closely attached to the stomach wall, and negative pressure inhalation not only makes the patient very uncomfortable but also causes nausea and vomiting. The patient will be able to get out of bed because the nasogastric tube is difficult to get out of bed, which plays a role in intestinal function rehabilitation and psychological rehabilitation. Therefore, the nasogastric tube should be more suitable for placement. In the conventional treatment of gastrointestinal tumors, the catheter and the abdominal drainage tube are placed as usual. Place the drainage tube for two purposes: one is to discharge abnormal fluid in the body cavity; the other is common symptoms after drainage. The placement of the abdominal drainage tube not only does not reduce the possibility of anastomotic leakage but also affects the extra-bed activity in the early postoperative period and increases the abdominal area. The discomfort caused by the catheter is more intense. Many patients feel the strongest discomfort after anesthesia is not the discomfort caused by the knife but the discomfort caused by the catheter. Patients are always afflicted by it [5]. In addition to increasing the likelihood of bacterial infections in the urinary system, the catheter also moves early on the patient. Control surgical stress response, such as lateral incision, or use laparoscopic or hand-assisted laparoscopic surgery as much as possible. Compared with traditional open surgery, the secretion of stress-responsive hormone is not reduced in patients undergoing laparoscopic surgery, but the inflammatory response is significantly reduced. Laparoscopic surgery significantly reduces patient discomfort. Compared with traditional open surgery, laparoscopic surgery reduces the patient's stress response, significantly accelerates the patient's recovery, and shortens the length of hospital stay. Therefore, minimally invasive surgery is an important part of postoperative rapid rehabilitation surgery, which promotes the development of postoperative rapid rehabilitation surgery [6].

In addition to laparoscopic surgery, there are some minimally invasive surgical techniques for specific surgical procedures and standardized surgical techniques for mild tissue. A person's temperature below 36 degrees Celsius is too low. During operation, the operating room temperature is too low, the veins manage a large amount of cryogenic fluid, anesthesia caused by vasodilation, organ contact, or wounds, and other causes always cause the patient's hypothermia to be too low. Intraoperative hypothermia will increase the patient's stress response, allowing patients to recover quickly after surgery [7]. Lower body surface temperatures can cause many common symptoms, such as decreased liver metabolic rate, disordered blood clotting mechanisms, decreased immune function, increased likelihood of bacterial infection, and reduced drug metabolism, and may lead to severe heart and lung disease, which affect the prognosis of patients. That is to say, for gastrointestinal surgery, the patient is allowed to recover anal deflation and defecation after eating, for example, early intake of food can provide energy and nutritional support to the patient before eating. It also reduces the likelihood of matching leaks in the abdominal cavity, bacterial infections in the incision, residual bacterial infections, and abdominal abscesses. The principle of small batches and increments can be followed multiple times. It allows patients to eat a certain amount of liquid food within 12 hours after surgery, such as no gastrointestinal discomfort. The normal diet can be resumed 24 hours after surgery, and intravenous medication is stopped. Nutritional foods can also be taken orally within 4 days after surgery to meet the patient's energy and protein intake and increase daily intake after surgery. Due to research quality issues, not all relevant data can be directly applied to clinical care work. The basics of all relevant data require scientific and effective analysis, evaluation, and screening of clinical nurses. Only in this way can we obtain the most authentic and reliable research basis, and the basis obtained can be used to solve this problem [8].

Scholars such as Tsang found that clinical practical problems have improved the scientific nature of clinical decision-making and improved the overall quality of clinical care services. At present, the ability of clinical nurses to evaluate evidence-based nursing medicine and its application in evidence-based nursing medicine is not very satisfactory. Clinical nutritional support is complex and has many symptoms. In the course of pharmacy care, nutrition evaluation should be carried out according to the specific conditions of patients. This requires clinical pharmacists to use their expertise and appropriate nutrition screening tools to determine the patient's nutritional status and whether nutritional support and nutritional screening tools are needed. Choose the appropriate nutritional prescription [9]. Tahan and other scholars explored the nutritional model based on the indicated parenteral nutrition. The foreign standard parenteral nutrition index is used as long as the gastrointestinal tract has function, but in China, not only the gastrointestinal function but also ensure the safe use of enteral nutrition. This is also why the proportion of parenteral nutrition is too high before the prescription. Clinical pharmacists should control the indications according to national guidelines and clinical patients' own conditions and follow the guidelines but not always follow the standard for pharmacy services. Third, clinical pharmacists should properly monitor and advise on the process, dosage, and prescription of nutritional support. They should choose different nutritional prescriptions according to the patient's height and weight according to the different conditions of the disease, so as to achieve the actual use of the drug. In addition, the rate of administration is a key component of observation. Different speeds can lead to different clinical outcomes. Fourth, the choice of the appropriate route of administration depends on whether the patient uses enteral nutrition or parenteral nutrition before selecting the route of administration and then chooses oral, nasal feeding, stoma, peripheral vein, and central vein depending on the circumstances. Finally, when clinical pharmacists perform nutritional support, systematic evidence-based nursing education requires students' basic medical statistics, clinical epidemiology, related data searches, nursing research, and English. For example, without the previous courses, students are difficult to understand. Its concepts, principles, and methods have practical significance. As a result, many foreign universities offer more courses at the undergraduate level and above, especially at the graduate level [10].

This paper selects the clinical nurses of the three top three hospitals in a province as the research object, using the general data questionnaire, the general individual performance sensitivity scale, the evidence-based nursing application behavior questionnaire, and the evidence-based nursing application behavior willingness questionnaire, and the evaluation ability training needs questionnaire. Data collection was performed on 100 cases of gastrointestinal surgery clinical nurses. Analyze nurses' understanding of evidence-based nursing, the willingness of evidence-based nursing behavior, and the relevance of evidence-based nursing behaviors. Use multiple regression analysis methods to explore the influencing factors, and use statistical analysis of evidence-based nursing in the gastrointestinal surgery pipeline.

## 2. Proposed Method

### 2.1. Evidence-Based Nursing Medicine

Evidence-based nursing medicine is a relatively new concept of care with the development of evidence-based medicine. Its core idea is to apply the best contemporary evidence judiciously and unambiguously. It is not only an important part of evidence-based medicine but also a relatively new field of research. Based on the clinical experience of nursing, it is proposed that “evidence-based nursing medicine” is the most appropriate and has skilled clinical knowledge and experience and provide appropriate care according to the patient's wishes. The rules of clinical evidence-based care methods should include knowledge and skills based on clinical experience, patient needs, the most appropriate research basics, and available resources. It includes the following complete process: evidence-based difficulties, support, observe, understand, and apply. Identify suspected clinical experience and theory in the process of nursing clinical experience, discover evidence-based care laws to collect practical application data based on relatively reliable data sources, find the most appropriate care method, and then use a key from the perspective of whether it can achieve the most appropriate effect or whether it is needed. Evidence-based nursing contains three elements, these three elements must be organically combined to establish a correct concept, and nursing discipline can progress further research on its development and gradually cycle, continuous improvement, to achieve continuous improvement of the quality of effective care. Evidence-based nursing medical clinical experience brings nursing science into a new era. Combine nursing research with clinical care experience to make mathematical medicine truly entered the era of research disciplines.

The application of evidence-based nursing medicine to nursing staff should follow the following five specific steps: The first step is to clarify the problems in clinical experience, that is, to ask questions and to find out the problems that patients need to solve by evaluating the application of thinking methods; the second step is to find relevant care information, that is, collect relevant information. In the third step, according to the epidemiological discipline and the evidence-based medical evaluation rules, the basic research is strictly evaluated, and the authenticity and reliability of the relevant data are found. The fourth step is to apply the most suitable basic examples. Guide the clinical method, that is, develop the nursing method according to the clinical relevant professional knowledge and the actual situation of the patient; the fifth step: evaluate the nursing effect and efficiency according to the clinical experience and closely observe and scientifically evaluate the basic effect in the application process. Therefore, we continue to summarize each experience and ultimately improve the academic level and quality of care of clinical nurses based on evidence-based clinical experience. Education must not only impart knowledge but also provide opportunities for students to innovate and learn independently. The environment should develop students' ability to acquire, apply, and innovate knowledge. In the teaching environment, students should change their learning concepts, use questionable thinking methods, seek practical application of existing clinical experience rules, and continuously improve the quality of care in future clinical nursing experience. In order to cultivate students' clinical thinking ability and medical ethics in medical teaching, students should pay attention to practical operation and ensure the accuracy and standardization of operation. With the emergence and development of society, the lack of medical and health resources, the rising cost of medical and health services, and the increase in demand have become global issues. This is due to the continuous expansion of the population base. Therefore, the most important thing is to promote the scientific and appropriate clinical methods of medical staff to promote a better clinical experience. The results of foreign medical education research show that the clinical experience and behavior of clinicians are affected by many factors. Therefore, it is necessary to introduce the concepts and methods of evidence-based nursing medicine into education to adapt to future clinical experience. Evidence-based nursing education can reduce the feeling and distance between students and practice and can more effectively promote students to understand and use knowledge.

### 2.2. Evidence-Based Nursing Skills and Behavior

Evidence-based nursing is a scientific research that is based on the problem (requires nurses to have scientific research capabilities and translate application problems into theoretical problems). Through the essence of evidence-based nursing knowledge, nurses are required to use epidemiological statistical knowledge as a link to evaluate, select evidence, and acquire knowledge in English to obtain the latest information. Evidence-based nursing knowledge emphasizes clinical practice as the starting point, combining scientific research theory with clinical expertise and experience and patient needs. With new and best “bases”, use supplemental information, “specific clinical issues,” to sample some of the data and validate and enrich the best empirical evidence for clinical problem resolution. Through this way of thinking, it is possible to present the specific steps and processes of evidence-based nursing medical knowledge, evidence-based methods, or evidence-based nursing medicine, as well as the knowledge content and ways of thinking involved in the main steps, including nurses' evidence-based nursing medical basic knowledge, scientific research knowledge, epidemiological statistical knowledge, and English knowledge, reflecting nurses' evidence-based nursing medical knowledge ability from different aspects. Nursing majors cultivate basic knowledge of humanities and social sciences, medicine, preventive health care, and basic theoretical knowledge and skills of nursing. Evidence-based nursing medical skills were as follows: nurses must have relevant evidence-based skills to identify problems, find empirical evidence, and then use the best way to solve problems under the guidance of the correct way of thinking. Therefore, nurses are required to have the ability to select information sources, to assess the ability to discover information, to effectively use information to solve problems, to be proficient in identifying problems and clinical solutions, and to make decisions. The nurse's evidence-based nursing medical skills are reflected in different aspects. Evidence-based nursing attitude was as follows: it refers to the research and discussion of nursing staff on nursing theory knowledge, reflecting the attitude ability of nursing staff in evidence-based nursing medicine from different angles.

Evidence-based nursing medical behavior was as follows: Nursing staff should often develop positive habits, find relevant information and their professional knowledge, and better integrate the useful research results of the application to solve clinical application problems, mainly reflected in how to obtain evidence-based applications. Basic or guidelines related to the program and solve application problems were as follows. Evidence-based nursing medicine requires modern nurses to have a knowledge structure systematically and modernize knowledge with the depth of professional basic theory and the breadth of relevant disciplines. Only by getting into the understanding of its connotation and basic steps, as well as its meaning and meaning, we combine the theory and knowledge with our common knowledge and effective methods and apply one theory to the specific clinical work. Clinical nurses have basic knowledge and relevant knowledge of evidence-based nursing medicine. Evidence-based nursing medicine focuses on utilizing the best basics available. The best research is basically obtained through scientific clinical research results and verified in clinical applications. Nurses are required to have strong scientific research knowledge and ability to continuously produce new research results. At the same time, when applying evidence-based medicine, nurses must not only use evidence but also learn to study and evaluate it, evaluate whether it is really suitable for the corresponding patients, and use it flexibly. This requires nurses to have clinical knowledge of epidemics and face bedside epidemics. Disease research methods can provide an effective external basis for evidence-based nursing medicine; on the other hand, in the face of bed-related epidemiological critical judgment methods, clinical nurses can more effectively select science from a large number of relevant data. Effective external evidence is based on clinical decision-making. Syndicated nursing medicine is basic. On the other hand, mastering statistical knowledge can help clinical nurses to basically identify the abuse of statistical processing and improve the reliability of systematic evaluation in evidence-based applications. In addition, ANOVA and regression analysis in mathematics are also beneficial for analyzing medical data and making inferences.

As the link between medical technology and information dissemination, medical English plays an important role in the introduction of evidence-based nursing medicine. It has a direct impact on learning the advanced experience of international evidence-based nursing medicine. An important reason for medical nursing technology methodology is that nurses are required to have a strong ability to read English in order to achieve the “latest and best evidence” required for the application of evidence-based nursing medicine. Good evidence-based nursing medical skills are key to improving the ability of evidence-based nursing medicine. Nurses must have relevant evidence-based skills in order to identify problems, find empirical evidence, and then use the best methods to solve problems under the guidance of the correct way of thinking. Information ability refers to the ability to select information sources, evaluate and discover information, and effectively use information to solve problems when determining information needs. Information ability is the foundation of development and creation, it is helpful to people's success, and it is the key to distinguish modern talents from traditional talents, mainly in the use of relevant data and search tools, the use of nursing database and Internet query nursing research results, the correct evaluation of nursing professional data, and the ability to find relevant research to solve problems encountered in clinical applications. Critical thinking ability refers to more appropriate questions, good at finding problems, and scientifically solving nursing problems. It can help nurses develop skills and apply the skills necessary for evidence-based nursing medicine, mainly reflected in the ability to find problems, solve clinical problems, and make decisions. Evidence-based attitude refers to the cognition of evidence-based nursing medicine and the behavioral tendency of evidence-based nursing medicine. A correct understanding and positive attitude towards evidence-based nursing medicine is the initiator of evidence-based care applications.

It includes the value orientation and acceptance of evidence-based applications. An excellent nursing worker not only needs solid evidence-based nursing knowledge and active evidence-based nursing attitude but also needs solid evidence-based nursing application behavior. Behavior is fundamental to the effectiveness of all good applications, because with the reform of the medical system, research is very important for nurses. Nursing staff should develop the habit of actively and regularly searching for relevant information, better integrate professional knowledge, and use the useful information obtained to ensure certainty.

### 2.3. Influencing Factors of Evidence-Based Nursing Medicine

Evidence-based nursing medical behavior is mainly how to actively obtain relevant evidence-based application and solve problems in application. The nurse did not understand the results of the study; the nurse did not believe the results; the nurse did not know how to use the findings. At the same time, the results of nurses' applied research are related to their ability to receive education. The higher the level of nurse education, the better the effect of applied research. Therefore, if these constraints can significantly affect the basic ability of nursing staff to apply evidence-based nursing medicine, the goal of transforming research results into economic benefits and social benefits can be achieved, thereby improving the quality of care. This may be related to the training objectives of nursing education at different levels of education. Undergraduate nursing students have more opportunities to acquire new knowledge and concepts, such as evidence-based nursing medicine, and to obtain broader and in-depth information. Education is also one of the reasons for evidence-based cognition of clinical nurses. The level of evidence-based nursing medical knowledge of general undergraduate nursing staff is higher than that of self-study undergraduate or network undergraduate nursing staff. There was no statistical difference in the level of evidence-based knowledge between general undergraduate nursing students and middle nursing students. The general undergraduate nursing program is more comprehensive and has a wider range of knowledge. This may be due to the fact that the current secondary vocational education is positioned as a skill-based and service-oriented talent. Even if they obtained a bachelor's degree in the later period, they have more theoretical knowledge, but they are subject to past educational experience. Therefore, they cannot be covered and imprisoned by past experiences, and they should strive to pursue new life experiences and do not let past experiences limit future possibilities. The goal of the work is to directly carry out specific steps in the application of care, and there is a lack of questionable thinking in research. At the same time, this difference in attitudes and beliefs may further influence their enthusiasm and enthusiasm for evidence-based nursing medicine in clinical work. The evidence-based cognitive level of general undergraduate nursing staff is higher than that of self-study undergraduate nursing staff. From the influence of learning forms on evidence-based knowledge and attitudes, it can be seen that ordinary undergraduate nursing students have certain advantages in evidence-based knowledge and skills, evidence-based attitudes, and belief levels: the higher the level of evidence-based knowledge of nursing students participating in evidence-based applications. It can be seen that evidence-based knowledge learning promotes the development of evidence-based applications, and evidence-based application behavior further promotes the ownership of evidence-based knowledge, which is interrelated, mutually reinforcing, and jointly improved. Learning evidence-based nursing medicine in clinical applications is also an evidence-based learning method that college students expect. In the future, the evidence-based concepts and skills of clinical nurses should be strengthened. Through oral and individual teaching, nursing students should gradually learn and master evidence-based knowledge and skills and form behaviors that actively use evidence-based concepts and skills in practical work.

One of the core elements of evidence-based care medicine is to consider the patient's subjective will. It also includes the most appropriate nursing research evidence available and the nursing staff's personal skills and clinical experience. For example, if care can play an “empathy” role, starting from the patient's actual preferences and trying to meet the patient's needs, the patient will eventually be satisfied, thereby improving the nurse-patient relationship. Evidence-based nursing physicians based on scientific rigorous research will improve the relationship between nurses and patients. Research and application work itself is more conducive to the health of patients. Some people may not have an in-depth understanding of the content of evidence-based nursing medicine. Especially when considering the subjective will of the patient, it is often easy to ignore the content when applying evidence-based applications. Part of the motivation for learning is mainly to complete the learning task and lack of active exploration and experiment in the learning process, which may be limited by the fixed thinking mode in school education. This will cause students to become less and less interested in learning and even have a mentality of learning weariness. In addition, because the nursing nurse works under the guidance of the teacher, the nursing behavior is mainly based on the teacher's behavior, and there is no clinical decision-making power. Clinical decision-making is not just a unilateral event of physicians and must be fully coordinated with patients and families to truly make medical decisions. At this stage, the cognitive rate of evidence-based nursing staff is low, and the application model of evidence-based nursing also hinders the development of evidence-based application behavior of nursing students. Evidence-based nursing medicine requires existing nursing knowledge to keep pace with the times. This requires the idea of lifelong learning. After graduating, they can insist on in-depth exploration of their professional knowledge when they are engaged in practical work. At this time, the autonomous learning method characterized by self-diagnosis, self-planning, and self-learning is more satisfactory, which meets their learning needs. The characteristics of the nursing discipline determine the value of qualitative research. Especially in the field related to human response and consciousness, qualitative research is more meaningful than quantitative research, which can further strengthen the evidence-based ability and ability training of clinical nursing teachers, and help students gradually learn and master evidence-based knowledge and skills through vocabulary and examples. At the same time, teachers and students can work together to find the best query basis, and in combination with the actual working environment and patient needs, and carefully and clearly applied to clinical work to improve the quality of care services.

## 3. Experiments

### 3.1. Experimental Settings

1. In order to ensure the fairness and justice of the experiment and the reliability of the data, the subjects selected 100 patients and nurses who met the inclusion criteria and underwent surgery in the gastrointestinal surgery wards of three tertiary hospitals in a province
2. The standard patients are older than or equal to 18 years old, less than or equal to 70 years old, hospitalized for surgery, need pipeline care, have smart phones, and will use WeChat function, voluntarily participate, and sign informed consent and patient supervision

### 3.2. Experimental Methods

1. Presurvey: according to relevant data, the presurvey sample size is more than 50 cases. In this study, 80 nurses were selected from different levels of nurses. Considering the questionnaire's response rate and other issues, the sample size was appropriately expanded. Preinvestigation can include controversial issues in the plan, in order to demonstrate the design from a clinical perspective, eliminate doubts, and further formulate a reasonable and feasible clinical investigation plan
2. Cross-sectional survey (the descriptive data obtained were collected at a certain point in time or within a short period of time): more than 90 nurses were randomly selected from the ward. Considering the problems such as the recovery rate of the questionnaire, the sample size is appropriately expanded; so, the sample size of this study is set to 100. The single analysis was as follows: the variance analysis method was used to compare the basic ability of evidence-based nursing and the total score of knowledge dimension; the rank sum test method was used to compare the total scores of empirical skills, attitudes, and behavioral dimensions (deviated distribution measurement data). Multivariate analysis method was as follows: the multiple regression analysis method was used to screen the causes of the impact of evidence-based nursing medical ability on nurses from the four dimensions of evidence-based nursing medical ability and evidence-based nursing medical ability. Canonical correlation was as follows: a typical correlation analysis method was used to analyze the correlation between the two groups of variables and the nurses' evidence-based nursing medical ability. Questionnaire reliability and validity analysis method were as follows: according to the degree of relevance of the questionnaire components and expert description content, the surface validity of the questionnaire was evaluated, and the structural validity of the questionnaire was evaluated by the factor analysis method. The analysis of variance was used to analyze the validity of the questionnaire. Evidence-based ability and its validity were analyzed for differential validity, and questionnaires were conducted. The internal reliability of the volume was as follows: on-site investigation, organization, interpretation, guidance, and recycling inspection. Filter out the abandoned questionnaires, determine the criteria for the valid questionnaire, check the validity of the questionnaire one by one before entering, and record the number of the invalid questionnaire

## 4. Discussion

### 4.1. Respondents' Knowledge of Evidence-Based Medicine

#### 4.1.1. Evidence-Based Medicine to Understand the Population Comparison

According to the statistical data analysis as shown in Figure 1 and Table 1, there are more gender surveys on evidence-based medicine, and 23 respondents believe that evidence-based medicine men know more; 45 respondents believe that evidence-based medicine women are more understanding; the other 32 respondents believe that the understanding of evidence-based medicine is “no gender difference.” Of the ages with more knowledge about evidence-based medicine, 11 respondents chose “unclear.” 70 respondents selected “youth.” 10 respondents chose “middle-age.” 8 were interviewed. The person selected “old age,” and one respondent selected “no age difference.”

#### 4.1.2. Analysis of the Clinical Knowledge of Evidence-Based Nursing with Different Academic Qualifications

According to the data analysis, as shown in Figure 2, the undergraduate knowledge of the clinical knowledge and skills of evidence-based nursing medicine is far more than the knowledge of the clinical skills of the nurses who graduated from the college. Because undergraduate nurses have a more positive perception of evidence-based nursing, they believe that evidence-based nursing is important to nursing practice and quality. The respondents understand the meaning and significance of evidence-based nursing. It is generally more than the background and steps for evidence-based care.

### 4.2. Evidence-Based Medicine for Gastrointestinal Surgery Pipeline Nursing Analysis

#### 4.2.1. Respondents' Understanding of Gastrointestinal Surgery Pipeline Care

According to the data analysis, according to the data analysis, as shown in Figure 3 and Table 2, the respondents' understanding is as follows: “unclear” respondents have 9; “learn more” respondents have 65 bit. There are 26 respondents who “learn less.” Most of the respondents know more about evidence-based medicine in gastrointestinal surgical tubing care.

#### 4.2.2. Analysis of the Application Effect of Gastrointestinal Surgery Pipeline Nursing

According to the data analysis, as shown in Figure 4, the application of evidence-based medicine for gastrointestinal surgery pipeline nursing is as good as 80%, and the application of evidence-based medicine for gastrointestinal surgery pipeline care is not good, up to 12%, based on evidence-based medicine. The gastrointestinal surgery pipeline care application effect is not obvious at 8%.

## 5. Conclusions

1. The interaction between individual performance, evidence-based nursing medical application experience and training experience is an important reason for clinical nurses' evaluation ability. The clinical nurses in the top three hospitals have higher requirements for training based on assessment ability, which is why the clinical nurses in the top three hospitals have higher requirements for training based on assessment ability. Under this circumstance, the nurses with higher training requirements are basically more in the early stage, that is, nurses who have basically high evaluation ability can be trained in advance. The nurses are all trained. Managers generally have a positive attitude towards evidence-based nursing medicine. The younger the working life, the more positive the attitude of nurses to evidence-based nursing; the evidence-based skills and behavioral level are good; evidence-based nursing medicine breaks the traditional way of thinking and working mode. This is the basicity of compliance, requiring clinical care to be basically demonstrated in strict scientific facts
2. Ways to acquire professional knowledge, solve clinical practical problems, and develop nursing methods. Nursing students mainly rely on professional books and senior nurses, and the opportunity to apply evidence-based nursing medicine is almost zero, which indicates that clinical knowledge is mainly from personal clinical experience. Teaching nursing students or senior nurses. Clinical teachers do not have the ability to actively improve new knowledge to understand the frontiers of nursing development and update existing knowledge. Some inefficient specific steps can also be replaced by specific steps that are proven to be more effective to improve the ability of nursing research staff and care applicants in evidence-based care medicine. Evidence-based nursing medicine capabilities mainly include knowledge integration ability and knowledge application ability. Strengthen the awareness of evidence-based application of nursing staff, and promote the positive, active and full use of basic resources by clinical front-line staff to improve the knowledge application ability of clinical employees. For the systematic education and training of evidence-based application in the later stage, it lays a foundation for cultivating clinical nursing talents with evidence-based nursing medicine ability. Promote the development of evidence-based nursing medicine applications. The application of evidence-based nursing medicine can effectively promote the transformation of nursing knowledge and research results into clinical applications. However, the application of evidence-based nursing medicine is a systematic and complex project involving a wide range of fields that requires a unified understanding and collaboration between decision makers, managers and applicants
3. The ideological center of evidence-based nursing medicine is to provide services to customers by using the latest and best scientific evidence. This affects experiential and intuitive care that has long been embedded in nurses and used by nurses. This has made evidence-based nursing medicine a far-reaching impact on nursing disciplines, patients, health care and society. Evidence-based nursing medicine organically combines nursing research and nursing applications, making nursing truly a research-oriented profession, supporting nurses to further seek professional autonomy and autonomy. The concept of evidence-based nursing medicine is a combination of science and technology. It requires medical staff to consider medical costs when developing and implementing a medical plan, and to control the rapid growth of medical expenses

## Figures and Tables

**Figure 1:** Age survey on evidence-based medicine.

**Figure 2:** Clinical understanding of evidence-based nursing with different education.

**Figure 3:** Understanding of nursing of gastrointestinal operation pipeline in evidence-based medicine.

**Figure 4:** Nursing effect of gastrointestinal operation pipeline.

**Table 1:** Gender survey on knowledge of evidence-based medicine.

Male	23%
Female sex	45%
No gender difference	32%

**Table 2:** Understanding of nursing of gastrointestinal operation pipeline in evidence-based medicine.

Unclear	9%
Know more	65%
Less understanding	26%

## Data Availability

No data were used to support this study.
